# Effect Evaluation of Norepinephrine on Cardiac Function in Patients with Sepsis by Cardiac Ultrasound Imaging

**DOI:** 10.1155/2022/5896791

**Published:** 2022-06-20

**Authors:** Wei Zhou, Yuyu Li, Baocheng Yang, Xianjun Wang

**Affiliations:** Department of Emergency Medicine, The First People's Hospital of Lianyungang, The First Affiliated Hospital of Kangda College of Nanjing Medical University, Xuzhou Medical University Affiliated Hospital of Lianyungang, Lianyungang, 222000 Jiangsu, China

## Abstract

In order to investigate the therapeutic effect of norepinephrine on patients with sepsis and the effect of echocardiography on the diagnosis of cardiac function in patients with sepsis, 86 patients with sepsis were selected as research objects and randomly divided into two groups. Patients in the control group (*N* = 43 cases) received conventional treatment (1~15 *μ*g/kg∗min dopamine), and those in the experimental group (*N* = 43 cases) received conventional treatment+norepinephrine therapy (0.05~0.5 *μ*g∗kg^−1^/min). The clinical efficacy, cardiac ultrasonography results, and hemodynamic indexes of patients between the two groups were analyzed and compared. The results showed that the total effective rate of treatment in the experimental group (97.7%) was significantly higher than that in the control group (81.4%) (*P* < 0.05). The maximum, minimum, and average values of mitral valve E peak flow velocity (VEpeak) and left ventricular outflow tract peak flow velocity (Vpeak), respiratory variability of mitral valve E peak flow velocity (*Δ*VEpeak), and respiratory variability of peak flow velocity (*Δ*Vpeak) were all significantly greater than those of the control group (*P* < 0.05). The area under the receiver operating characteristic curve (AUC) of *Δ*VEpeak and *Δ*Vpeak for predicting positive volume response in patients with sepsis was 0.934 and 0.913, respectively; the sensitivity was 0.828 and 0.827; the specificity was 0.936 and 0.893; and the Youden indices were 0.765 and 0.712, respectively. In short, norepinephrine had a high total response rate in patients with sepsis, and echocardiography can well evaluate the effect of norepinephrine on cardiac function in patients with sepsis, which is worthy of further promotion.

## 1. Introduction

Sepsis is a systemic inflammatory response caused by the dysregulation of the body's immune response triggered by infectious factors, which may lead to multiple organ dysfunction and be life-threatening [1]. Globally, 19 million people suffer from sepsis every year, and one-quarter or more of them die, and the incidence of sepsis is increasing year by year with the aging of the population [2]. In clinical practice, patients with sepsis are usually divided into sepsis, severe sepsis (sepsis with acute organ dysfunction and hypotension), and septic shock (sepsis with hyperlactatemia or persistent hypotension that is difficult to correct with fluid resuscitation). The above classification is of great significance for judging the prognosis and severity of sepsis [3, 4]. During the development of sepsis, the primary infection site may be involved, and it may involve important organs of the body in severe cases, such as the heart, lungs, and liver. The etiology of sepsis is clear and is caused by severe infection of the body [5]. Pulmonary infections are the most common cause of patients with sepsis, accounting for more than 50% of all sepsis, followed by abdominal and urinary tract infections [6].

Sepsis is an acute and critical illness that requires early identification and early intervention to save patients' lives to the greatest extent and improve prognosis. At present, the examination methods for sepsis include blood test, urine culture test, wound secretion test, respiratory secretion test, and imaging test (including CT, ultrasound, and nuclear magnetic resonance) [7, 8]. Echocardiography in patients with sepsis usually shows decreased left ventricular systolic function and left ventricular dilation and can also present with left ventricular diastolic dysfunction. If the mitral valve annular blood flow velocity decreases, it indicates that the left ventricle has diastolic dysfunction, and the presence of left ventricular diastolic dysfunction indicates that the patient is seriously ill. In addition to affecting the left ventricle, septic cardiomyopathy also affects the right ventricular system, usually due to cardiac afterload [9, 10].

The common clinical treatments for sepsis include drug therapy and surgical therapy, in which antibiotics, low-dose glucocorticoids, insulin, painkillers, and analgesics are widely used [11]. The main purpose of vasoactivating drugs in the treatment of sepsis is maintaining blood pressure, maintaining the blood supply of the heart and brain and other important organs, and reducing the mortality rate. Both norepinephrine and dopamine have been used as important vasopressors for patients with septic shock [12]. Studies revealed that norepinephrine can significantly increase systemic vascular resistance and mean arterial pressure (MAP) in patients with septic shock, with little change in heart rate, and is widely recognized as the drug of choice. Clinically, there has been some concern with the use of norepinephrine due to its properties of constricting renal perfusion vessels. However, due to its ability to increase renal blood flow by providing higher perfusion pressure, patients may have an increased glomerular filtration rate. It has been reported that immunosuppression is an intermediate factor between the severity of the disease and the adverse outcome of sepsis patients, and norepinephrine will drive the immunosuppression response of sepsis patients, thus playing a role in regulating the immune defense of the host [13]. In recent years, studies on the efficacy of norepinephrine in the clinical treatment of patients with sepsis have emerged in an endless stream [14, 15], but there are few studies on the cardiac ultrasound and cardiac hemodynamics of patients with sepsis after norepinephrine treatment.

Therefore, this study was hoped to evaluate the influence of norepinephrine treatment on cardiac function of patients with sepsis treated with antihypertensive drugs based on clinical cardiac ultrasound and hemodynamics. This study is aimed at providing some reference for clinical medication and cardiac function evaluation of patients with sepsis.

## 2. Materials and Methods

### 2.1. Research Objects

In this study, 86 patients with sepsis diagnosed in hospital from October 2017 to October 2020 were selected as the research objects. The age of the patients ranged from 19 to 78 years old; the mean age was 58.74 ± 12.85 years old, with 47 males and 39 females. The clinical diagnosis of sepsis was based on the 2016 edition of the Sepsis Rescue Campaign Guidelines (SSC) of the American Society of Critical Care Medicine and the European Society of Critical Care Medicine. If the Sequential Organ Failure Assessment (SOFA) score ≥ 2 points, it was the infection or suspected infection. All procedures of this work had been approved by the ethics committee of the hospital, and the subjects included had signed the informed consents.

The inclusion criteria of the patients were given as follows: (I) the patients met the diagnostic criteria for sepsis; (II) the patients were older than 18 years old; (III) the patients were unable to breathe spontaneously; and (IV) the patient was mechanically ventilated with an endotracheal tube due to respiratory failure. The exclusion criteria for patients were described as follows: (I) patients treated with norepinephrine for less than 24 hours; (II) patients with severe cardiovascular and cerebrovascular diseases; (III) patients with arrhythmia symptoms; and (IV) patients with contraindications to volume stress testing.

### 2.2. Grouping and Treatment

All patients with sepsis were randomly divided into two groups, with 43 cases in each group. Among them, patients in the control group were treated with conventional anti-infection methods, and the specific procedures were as follows. The patient's central venous pressure and invasive arterial pressure were firstly measured by central venipuncture, and then, the patient's blood uric acid and arterial blood gas were analyzed by urine output. In addition, 1 to 15 *μ*g/kg∗min of dopamine was adopted for anti-infective treatment.

On the basis of the basic treatment of the control group, the patients in the experimental group were treated with norepinephrine by 0.05~0.5 *μ*g∗kg^−1^/min. During this process, it was necessary to closely monitor the blood oxygen saturation, blood lactate, and other vital signs of patients. Anti-infective therapy was administered only once in both groups.

### 2.3. Volume Loading Test

Volume loading experiments were performed on both groups of patients [16]. In this experiment, all patients will be intravenously infused with 0.9% potassium chloride injection (30 min, 500 mL) through the peripheral veins or central veins. Patients with pulmonary edema complications should stop the infusion immediately. The stroke volume (SV) of the patient before and after the infusion was compared. If the difference was positive and the increase was more than 15%, the patient's volume loading test was positive and there was volume responsiveness. The calculation equation of SV difference ΔSV is shown in the following equation:

(1) $$\begin{array}{c} \Delta \text{SV}=\frac{{\text{SV}}_{2}-{\text{SV}}_{1}}{{\text{SV}}_{1}}\times 100\%. \end{array}$$

At the end of the volume stress test, the left ventricular outflow tract VTI, the maximum and minimum mitral valve E peak flow velocity, and the maximum and minimum LVOT peak flow velocity were measured again. It should calculate stroke volume (SV), mitral valve E peak flow respiratory variability, LVOT peak flow respiratory variability, etc.

### 2.4. Cardiac Ultrasonography and Detection Indicators

The cardiac ultrasonography equipment was used in this study. During ultrasonography to measure stroke volume, the patient was placed in the left lateral decubitus position, and the cardiac probe was placed in the third or fourth intercostal space at the left sternal border. Its directional sign points to the patient's right shoulder, showing the parasternal long-axis view of the left ventricle, looking for the ultrasound image with the aortic valve open to the maximum, and measuring the left ventricular outflow tract (LVOT) diameter (*D*). The cardiac probe was placed at the apex of the heart to sample the apical four-chamber view and the apical five-chamber view. After that, the probe was placed under the aortic valve, pulsed Doppler (PW) sampling was performed, the left ventricular outflow tract spectrum was recorded, and the LVOT velocity time integral (VTI) was calculated.

When the mitral valve E peak flow velocity (VEpeak) and its respiratory variability (*Δ*VEpeak) and LVOT peak flow velocity (Vpeak) and its respiratory variability (*Δ*Vpeak) were measured by ultrasound, the cardiac probe was placed at the apex of the heart, and the marked point was facing the left shoulder. It could obtain the mitral valve orifice blood flow spectrum and the LVOT blood flow spectrum and measure the maximum and minimum values of mitral valve E peak flow velocity (VEpeak) and LVOT peak flow velocity (Vpeak). When the VEpeak, Vpeak, *Δ*VEpeak, and *Δ*Vpeak of patients were compared, the results of the volume stress test were undertaken as the gold standard to compare the differences of each index between the two groups of patients.

### 2.5. Summary of Clinical Indexes

During this work, the basic information of patients and various clinical indicators were collected. Basic information included age, gender, name, admission, and outpatient diagnosis, outcome, and treatment. Clinical index information included heart rate, blood pressure, blood routine, blood gas analysis, ventilator tidal volume, positive end-expiratory pressure, plateau pressure, Sequential Organ Failure Assessment (SOFA) score, and acute physiology and chronic health evaluation II (APACHE II) [17].

SOFA score is based on the total of respiratory, cardiovascular, liver, coagulation, kidney, and nervous systems. The scores range from 0 to 4, and the increase of the score reflects worsening organ dysfunction. Studies in the past 30 years suggested that SOFA scores can detect differences in disease severity and serve as an important evaluation standard for clinical studies. APACHE is the most widely used and authoritative scoring method to evaluate the severity and prognosis of all kinds of critically ill patients. The APACHE II score consists of three parts, namely, acute physiological score, age score, and chronic health score.

### 2.6. Evaluation of Ultrasound Diagnosis Effect

In this work, *Δ*VEpeak and *Δ*Vpeak in echocardiography of two groups of patients were measured. Receiver operating characteristic curve (ROC) and area under the ROC (AUC) were used to predict the predictive power of patients with sepsis volume responsiveness in evaluating the effect of norepinephrine treatment. In addition, accuracy, sensitivity, and specificity of echocardiography diagnosis were calculated.

(2) $$\begin{array}{c} \text{Accuracy}=\frac{A+D}{A+B+C+D}\times 100\%,\\ \text{Sensitivity}=\frac{A}{A+C}\times 100\%,\\ \text{Specificity}=\frac{D}{B+D}\times 100\%. \end{array}$$

In the above equations, *A*, *B*, *C*, and *D* represented true-positive results, false-positive results, false-negative results, and false-positive results, respectively.

### 2.7. Statistical Methods

Statistical software SPSS19.0 was used to process the experimental data. The measurement data were expressed as mean ± standard deviation ($\bar{x}\pm \text{s}$), the mean comparison between groups was by *t* test, the enumeration data was expressed by percentage (%), and the *χ*^2^ test was used. *P* < 0.05 indicated that the difference was statistically significant.

## 3. Results

### 3.1. General Information

Figure 1 was a comparison chart of the general data of the two groups of patients. As illustrated in the figure, there were 25 males and 18 females in the experimental group, with an average age of 57.83 ± 13.43 years old and an average heart rate of 92.54 ± 11.32 beats/min. There were 22 males and 21 females in the control group, with an average age of 59.02 ± 12.41 years old, and the average heart rate was 93.03 ± 10.89 beats/min. After comparison, the ratio of males and females, average age, and average heart rate between the two groups were significantly different (*P* < 0.05). In addition, comparison on the etiology of sepsis between the two groups revealed that there were 24 cases of pulmonary infection, 8 cases of abdominal infection, 4 cases of bloodstream infection, and 29 cases of septic shock in the experimental group. In the control group, there were 25 cases of pulmonary infection, 7 cases of abdominal infection, 5 cases of bloodstream infection, and 28 cases of septic shock. There was no significant difference in the etiology distribution between the two groups (*P* > 0.05).

### 3.2. Comparison of Clinical Efficacy between Two Groups

Figure 2 shows a comparison chart of the clinical efficacy of the two groups of patients. As illustrated in Figure 2, 36 cases in the experimental group were markedly effective, 6 cases were effective, and 1 case was ineffective, with a total effective rate of 97.7%. In the control group, 24 cases were markedly effective, 11 cases were effective, and 8 cases were ineffective, with a total effective rate of 81.4%. After comparison, it was found that the total effective rate of treatment of patients in the experimental group was significantly higher than that in the control group, and the difference was statistically significant (*P* < 0.05).

Figure 3 shows a comparison chart of the APACHE II score and SOFA score of the two groups of patients. As demonstrated in the figure, the APACHE II score and SOFA score of the experimental group were 14.2 ± 4.6 and 15.9 ± 3.9, respectively, while the APACHE II and SOFA scores of the control group were 18.3 ± 5.9 and 17.5 ± 4.3, respectively. After comparison, it was found that the APACHE II score and SOFA score of the experimental group were significantly lower than those of the control group, and the differences were statistically significant (*P* < 0.05).

### 3.3. Echocardiography of Patients

Figure 4 shows the echocardiography diagram of some patients. Patients with sepsis echocardiography showed that the atria and ventricles were enlarged to varying degrees, the mitral and tricuspid valves and/or the aorta were refluxed, and symptoms of pulmonary hypertension of varying degrees were present.

### 3.4. Echocardiographic Hemodynamic Results of Two Groups

Figure 5 shows the comparison of the maximum, minimum, and average values of VEpeak and Vpeak between the two groups.  Figure 6 shows the comparison of *Δ*VEpeak and *Δ*Vpeak between the two groups. Figure 5 shows that the maximum, minimum, and average values of VEpeak in the experimental group were 94.34 ± 16.41 cm/s, 78.98 ± 13.72 cm/s, and 87.35 ± 15.22 cm/s, respectively. They were significantly higher than those in the control group (87.43 ± 18.42 cm/s, 69.12 ± 16.43 cm/s, and 74.76 ± 17.41 cm/s), and the difference was statistically significant (*P* < 0.05). The maximum, minimum, and average values of Vpeak were 92.87 ± 12.92 cm/s, 82.15 ± 14.10 cm/s, and 87.23 ± 14.92 cm/s, respectively. Compared with those of the control group (86.47 ± 16.76 cm/s, 75.73 ± 16.43 cm/s, and 81.44 ± 17.41 cm/s), the difference was statistically significant (*P* < 0.05).  Figure 6 shows that *Δ*VEpeak and *Δ*Vpeak in the experimental group were 0.18 ± 0.07 and 0.12 ± 0.05, respectively, which were significantly higher than those in control group (0.13 ± 0.08 and 0.08 ± 0.03), with statistically significant differences (*P* < 0.05).

### 3.5. Evaluation of the Predictive Value of Echocardiography in Patients

Figure 7 shows the ROC curve of *Δ*VEpeak and *Δ*Vpeak predicting positive volume response, and Figure 8 shows the prediction accuracy result obtained according to Figure 7. It can be known from Figures 7 and 8 that the AUCs of *Δ*VEpeak and *Δ*Vpeak in patients with sepsis for predicting positive volume response were 0.934 and 0.913, respectively; the sensitivity was 0.828 and 0.827; the specificity was 0.936 and 0.893; and Youden indices were 0.765 and 0.712, respectively.

## 4. Discussion

The incidence of sepsis is high. There are more than 18 million cases of severe sepsis in the world each year, there are 750,000 patients with sepsis in the United States each year, and this number is also increasing at a rate of 1.5% to 8.0% per year [18]. Sepsis is a dangerous condition with a high fatality rate, with approximately 14,000 deaths per day from its complications worldwide and approximately 215,000 deaths per year in the United States [19]. According to foreign epidemiological surveys, sepsis has become the main cause of death in noncardiac patients in intensive care units, and its fatality rate has exceeded myocardial infarction [20]. Current research suggests that the disease development process of sepsis involves systemic inflammatory network effects, gene polymorphisms, immune dysfunction, abnormal coagulation function, tissue damage, and abnormal host responses to different infectious pathogenic microorganisms and their toxins. It is closely related to the pathophysiological changes of the multisystem and multiorgan of the body [21].

By comparing the prognostic effect of patients with sepsis treated with conventional treatment and norepinephrine, it was found that the total effective rate of patients treated with norepinephrine in the experimental group was significantly higher than that in the control group, and the difference was statistically significant (*P* < 0.05). In addition, the APACHE II score and SOFA score in the experimental group were significantly lower than those in the control group, with statistically significant differences (*P* < 0.05), which was consistent with the study of Zhou et al. [16]. These results indicated that norepinephrine treatment had a significant effect on patients with sepsis, which can significantly relieve the degree of organ failure in patients with sepsis and improve the prognosis and health of patients. In sepsis, due to abnormal vasoconstriction and diastolic function and increased permeability, the body has decreased blood volume and hypoperfusion of tissues and organs in the early stage, so timely effective fluid resuscitation has become a key measure for the treatment of sepsis [22]. If fluid resuscitation does not improve the patient's blood pressure and organ hypoperfusion status, vasoactive drugs should be given. If the patient is facing life-threatening shock, even if the hypovolemia is not corrected, it should be given at this time. However, norepinephrine, as a common hypertensive drug in clinical practice, has been proved to have good vascular activation effect on patients with septic shock [23].

Echocardiography in patients with sepsis usually shows decreased left ventricular systolic function, left ventricular dilation, and left ventricular diastolic dysfunction. Usually, it is accompanied by a decline in left ventricular ejection fraction (LVEF), and the blood flow velocity of the annulus of the mitral and aortic valves decreases, resulting in blood reflux of varying degrees. Sepsis cardiomyopathy involves not only the left ventricle but also the right heart system, which is usually caused by cardiac afterload [18].

The current early crystalloid solution and follow-up fluid therapy for sepsis can effectively promote the recovery of the patient's organ function and improve the patient's internal circulation. However, during use, it is necessary to repeatedly monitor the patient's hemodynamic status and continuously optimize the titration cycle process of fluid therapy [24]. Among the noninvasive indicators of the cardiopulmonary interaction theory, the respiratory variability of the mitral valve E peak flow rate and the respiratory variability of the left ventricular outflow tract peak flow rate both study the respiratory variability of the arteriovenous vessels of the systemic circulation, which can well predict the internal blood flow of the heart. For respiratory variability volume responsiveness, mitral valve blood flow was the best predictor [25]. In this work, VEpeak, *Δ*VEpeak, Vpeak, and *Δ*Vpeak were used to evaluate the volume responsiveness of patients with sepsis and to compare the hemodynamic status presented by echocardiography in the two groups of patients after treatment. The results showed that the maximum, minimum, and average values of VEpeak and Vpeak, *Δ*VEpeak and *Δ*Vpeak in the experimental group were significantly greater than those in the control group, with significant differences (*P* < 0.05). The AUCs of *Δ*VEpeak and *Δ*Vpeak in patients with sepsis for predicting positive volume response were 0.934 and 0.913, respectively, the sensitivity was 0.828 and 0.827; the specificity was 0.936 and 0.893; and the Youden indices were 0.765 and 0.712, respectively. This shows that echocardiography performs well in evaluating cardiac function in patients with sepsis norepinephrine and has good predictive value.

## 5. Conclusion

In this study, the clinical efficacy and echocardiography of patients with sepsis treated with norepinephrine were analyzed, and it was found that the VEpeak and its respiratory variability rate and Vpeak index monitored by cardiac ultrasound can well monitor the cardiac function of patients with sepsis and have a high accuracy in evaluation of norepinephrine treatment. However, there were some shortcomings in this work. For example, the small sample size included in this work did not provide a detailed assessment of cardiac ultrasound in different types of patients with sepsis and the effect of norepinephrine treatment on cardiac functions of the patients. In the future, it is expected that further research will be conducted on the evaluation of echocardiography after norepinephrine treatment in different types of patients with sepsis. In conclusion, this work could provide a certain reference for the related research on the efficacy of vascular activating drugs and their effects on cardiac function in patients with sepsis.

## Figures and Tables

**Figure 1:** Comparison of general data of the two groups. (a) Shows the gender distribution diagram, (b) shows the comparison diagram of the average age, (c) shows the comparison diagram of the average heart rate, and (d) shows the distribution diagram of the etiology.

**Figure 2:** Comparison of clinical efficacy of two groups. (a) Shows the distribution diagram of the effective treatment; (b) shows the comparison diagram of the total effective rate of treatment. ^∗^Compared with the control group, *P* < 0.05.

**Figure 3:** Comparison of APACHE II score and SOFA score. ^∗^Compared with the control group, *P* < 0.05.

**Figure 4:** Echocardiography of patients. (a, b) Show the mitral valve regurgitation and regurgitation spectrograms of patients with sepsis with a small amount of mitral valve regurgitation, respectively; (c, d) show the spectrograms of aortic valve regurgitation and regurgitation in the apical five-chamber view of patients with sepsis with a small amount and moderate amount of aortic valve regurgitation, respectively; (e, f) show the images of mitral valve regurgitation in patients with sepsis with a small amount and moderate amount of mitral valve regurgitation, respectively; (g, h) show aortic valve regurgitation in patients with sepsis with a small amount and moderate amount of aortic valve regurgitation, respectively.

**Figure 5:** Comparison of the maximum, minimum, and average values of VEpeak and Vpeak. (a) Shows the comparison chart of the maximum, minimum, and average values of VEpeak; (b) shows the comparison chart of the maximum, minimum, and average values of Vpeak. ^∗^Compared with the control group, *P* < 0.05.

**Figure 6:** Comparison of *Δ*VEpeak and *Δ*Vpeak between the two groups. ^∗^Compared with the control group, *P* < 0.05.

**Figure 7:** ROC curve of *Δ*VEpeak and *Δ*Vpeak predicting positive volume response.

**Figure 8:** Prediction accuracy results of *Δ*VEpeak and *Δ*Vpeak in predicting positive volume response.

## Data Availability

The data used to support the findings of this study are available from the corresponding author upon request.
